This article has been retracted.

# HPV-16 Expression and Loss of Cell Differentiation in Primary Bladder Tumors

**DOI:** 10.1155/2022/6565620

**Published:** 2022-10-15

**Authors:** Lei Pang, Zijun Ding, Fei Li, Hongqiang Chai, Ming Wu, Jinkai Shao

**Affiliations:** ^1^Department of Urology, The Fifth Hospital of Shanxi Medical University (Shanxi Provincial People's Hospital), No. 29 Shuangta East Street, Yingze District, Taiyuan, Shanxi 030012, China; ^2^Department of Neonatology, Shanxi Children's Hospital, No. 13 North Xinmin Street, Xinghualing District, Taiyuan, Shanxi 030013, China

## Abstract

**Objective:**

Primary bladder tumors have a high degree of malignancy. To investigate the expression of human papillomavirus type 16 (HPV-16) in primary bladder tumors and the loss of cell differentiation and to explore the significance of HPV-16 detection, it is expected to be a disease. Treatment provides a theoretical basis.

**Methods:**

Fifty-seven patients with primary bladder tumors admitted to our hospital from January 2019 to January 2022 were selected as the research subjects, and they were divided into HPV-related groups according to the human papillomavirus (HPV) infection status (*n* = 28) and HPV unrelated group (*n* = 29). The general data of patients were collected, the expression of HPV-16 in bladder tissue samples was detected, and the correlation between pathological parameters and HPV-16 expression was analyzed.

**Results:**

Among HPV subtypes, HPV 16 subtype accounted for the highest proportion, followed by HPV-18 and HPV-6 subtypes; there was no significant difference in tumor stage (stage 1, stage a, stage 2a) between the HPV-related group and the HPV-unrelated group (stage 1, stage a, and stage 2a). *P* > 0.05); there was no significant difference in postoperative pathological expression (high expression and low expression) of patients (*P* > 0.05); there was no statistical difference in age and gender between HPV-related and HPV-unrelated groups (*P* > 0.05), HPV-related group and HPV-unrelated group compared daily regular drinking and smoking status, the difference was statistically significant (*P* < 0.05); HPV-16 expression was not correlated with tumor differentiation degree and age of patients (*P* > 0.05); the area under the curve (AUC) of HPV-16 for judging primary bladder tumor expression and cellular molecular deletion was 0.891, with a sensitivity of 83.94% and a specificity of 88.57%.

**Conclusion:**

HPV-16 is an upper, expressed in primary bladder tumors and will participate in the differentiation and loss of cells, which can provide effective guidance and basis for the diagnosis of primary bladder tumors, which is an important factor for judging the pathological stage and prognosis of patients and can provide a theoretical reference for the formulation of therapeutic measures.

## 1. Introduction

The latest reported data show that bladder tumor is a highly malignant tumor. In China, the incidence of bladder cancer ranks first in malignant tumors of the urinary system, and transitional cell carcinoma (TCC) accounts for about 90% of the pathological types of bladder tumors. However, the understanding of the pathogenesis of primary bladder tumors is low, and exposure to ionizing radiation, aromatic amines, and cyclophosphamide are currently identified as risk factors [1]. HPV mainly appears after tumor invasion, HPV infection can indirectly or directly cause human tumor formation, and in particular, can have an impact on pathological grade [2]. Before, HPV-16 fragment in bladder tissue was often detected by specific primer PcR. The results confirmed that there was a notable variation in the positive rate of HPV-16 fragment between normal bladder tissue and bladder tumor tissue. The expression of HPV-16 fragment in bladder tumor tissue was detected by Southemblot. The results showed that HPV-16 expression in bladder tumor was notably correlated with the occurrence of primary bladder tumor [3, 4]. At present, it is mainly treated by comprehensive treatment methods such as chemotherapy, immunotherapy, and photodynamic therapy. Benign bladder tumors can be cured after treatment, but malignant tumors are prone to recurrence and metastasis after treatment. For bladder cancer, the presence or absence of invasion is one of the important prognostic factors for bladder cancer. However, the premise of treatment is to analyze the factors affecting the disease literature and the expression of HPV-16 in order to have a better reference for disease treatment.

Based on this, 57 patients with primary bladder tumors admitted to our hospital between January 2019 and January 2022 were opted as the study subjects to preliminarily investigate HPV-16 expression and analyze the relationship with patient prognosis, hoping to provide morphological evidence for disease healing, as reported below.

## 2. Materials and Methods

### 2.1. General Data

Fifty-seven patients with primary bladder tumors admitted to our hospital from January 2019 to January 2022 were opted as the study subjects and divided into two clusters according to human papillomavirus (HPV) infection. HPV-related cluster (*n* = 28); 7 females; 21 males; aged 27-64 years; mean age (61.46 ± 3.58) years; HPV subtypes: HPV-6 : 3, HPV-16 : 8, HPV-18 : 5, HPV-26 : 1, HPV-39 : 2, HPV-45 : 1, HPV-51 : 1, HPV-53 : 2, HPV-56 : 1, HPV-59 : 1, HPV-66 : 1, HPV-68 : 1, and HPV-82 : 1; tumor stage: 9, stage a: 10, and stage 2a: 9; postoperative pathology: upper expression in 17 and bottom expression in 11. In the HPV-unrelated cluster (*n* = 29), there were 8 females and 21 males, aged 27–64 years, with a mean age of (63.10 ± 3.29) years; tumor stage: 8 situations of stage 1, 10 situations of stage a, and 11 situations of stage 2a; postoperative pathology: 7 situations of upper expression and 21 situations of bottom expression. This study has been approved by the ethics department, and patients are aware of the study.

*Inclusion criteria:* (1) HPV positive; (2) older than 18 years old; (3) cervical biopsy or staining pathology diagnosis [5], diagnosed as primary bladder tumor; (4) did not receive antitumor hormone intervention before the study; (5) good spirit; (6) life cycle more than 12 months.

*Exclusion criteria:* (1) infectious diseases; (2) immune diseases; (3) combined with bladder cancer outside the tumor; (4) bottom compliance; (5) organ damage; (6) lactating or pregnant women.

### 2.2. Methods

#### 2.2.1. Specimen Source

The specimens were opted from those who were pathologically diagnosed as primary bladder tumors. After the specimens were obtained, they were placed in EP tubes and then stored in -80°C refrigerator. Various data were collected from the patients, including age, gender, alcohol consumption, and smoking status.

#### 2.2.2. DNA Preparation and PCR Detection

*DNA sample extraction*: centrifuge the cell suspension, extract DNA, and perform various operations according to the kit instructions, then uniformly dilute the DNA concentration to 100 ng/*μ*L and store in -20°C equipment.

*Amplification PCR:* PCR amplification is performed using primer nucleotide sequences.

*PCR product electrophoresis:* agarose gel electrophoresis of PCR products, 10 *μ*L of PCR products were subjected to agarose gel electrophoresis (1.0%) and photographed by Tianneng gel imaging system.

*Judgment result:* if there is a bright band at the 217 bp position, and the prejudgment result is loaded at the same time, it is confirmed that the HPV-16 test is a positive result, and the product is analyzed by electrophoresis to verify the sequencing result.

### 2.3. Observation Indicators

*HPV subtype analysis of patients:* including HPV-6, HPV-16, HPV-18, HPV-26, HPV-39, HPV-45, HPV-51, HPV-53, HPV-56, HPV-59, HPV-66, HPV-68, HPV-82 HPV subtypes.

*Tumor staging:* count the number of situations of stage 1, stage a, and stage 2a, and calculate the proportion.

*Postoperative pathological expression:* count the number of situations with upper expression and bottom expression, and calculate the proportion.

*General information:* including age, gender, alcohol consumption (regular daily drinking, occasional/never), and smoking (smoking, quit smoking, never).

*Logistic regression analysis:* the correlation between HPV-16 expression and the degree of tumor differentiation and age of patients.

*The value of HPV-16 in judging the expression of primary bladder tumor and the value of cell and molecular deletion:* calculate the diagnostic sensitivity and specificity of HPV-16.

*Analysis of the prognosis of patients:* count the number of situations of single tumor and multiple tumors, count the number of patients with tumor-free survival, recurrence, and death, and calculate the proportion.

### 2.4. Statistical Methods

The count data was expressed as *n*(%), and the contrastion between clusters was performed by the *χ*^2^ test; the measurement data that obeyed the normal distribution was expressed as ($\bar{x}\pm s$), and the contrastion between multiple clusters was performed by one-way variance and repeated measures. The data were contrasted using the analysis of variance of repeated measures data, and *P* < 0.05 was regarded as a notable variation.

## 3. Results

### 3.1. Analysis of HPV Subtypes in Patients

Among HPV subtypes, HPV-16 subtypes accounted for the uppermost proportion, followed by HPV-18 and HPV-6 subtypes (Table 1 and Figure 1).

### 3.2. Tumor Stage Analysis of Two Clusters of Patients

None notable variation in tumor stage (stage 1, stage a, stage 2a) between the HPV-related cluster and the HPV-unrelated cluster (*P* > 0.05) (Table 2 and Figure 2).

### 3.3. Postoperative Pathological Expression Analysis of Two Clusters of Patients

None notable variation in postoperative pathological expression (upper expression and bottom expression) of patients (*P* > 0.05) (Table 3 and Figure 3).

### 3.4. General Data Analysis of Patients

None notable variation in age and gender between the HPV-related cluster and the HPV-unrelated cluster (*P* > 0.05). There was a notable variation between the HPV-related and HPV-unrelated clusters in daily regular drinking and smoking status (*P* < 0.05) (Table 4).

### 3.5. Correlation Analysis of HPV-16 Expression with Tumor Differentiation and Age in Patients

None correlation between the expression of HPV-16 and the degree of tumor differentiation and age of the patients (*P* > 0.05) (Table 5).

### 3.6. The Value of HPV-16 in Judging Primary Bladder Tumor Expression and Cell and Molecular Deletion

The area under the curve (AUC) of HPV-16 for judging primary bladder tumor expression and cellular molecular deletion was 0.891, with a sensitivity of 83.94% and a specificity of 88.57% (Figure 4).

### 3.7. Analysis of Patient Prognosis

57 patients, including 11 patients with single tumor and 46 patients with multiple tumors, were followed-up for 3 years. The follow-up found that 37 patients survived tumor-free, 17 patients recurred, and 3 patients died (Figure 5).

## 4. Discussion

Males aged 40-70 are the main cluster of primary bladder tumors, with invasive growth and papillary growth as the main growth patterns, and the results are in good agreement with the results of most domestic studies [6]. Regarding the correlation between bladder cancer and HPV, the research conclusions are controversial. Shaker et al. showed that the positive rate of high-risk HPV-16/18 in BUCC was significantly higher than that in chronic cystitis and normal bladder tissue, and it was related to the clinical staging of bladder cancer patients. There is a certain correlation. Polesel et al. detected HPV in urine, and the results showed that there was no significant correlation between HPV and bladder cancer. Schmid et al. conducted a prospective study on samples of Chinese and European populations, and the results showed that HPV infection was associated with the occurrence of bladder cancer. Not related to development. More and more studies have confirmed that patients with genitourinary tumors have a higher rate of HPV infection, especially HPV-16 infection [7, 8]. After the patient is infected, the P16 protein will be activated and overexpressed. It has a strong expression ability in the process of bladder tumor lesions and can judge the status of tumor lesions [9, 10].

Followed by HPV-18 and HPV-6 subtypes, no notable variation in tumor stage and pathological expression between the two clusters of patients, improving the comparability of the data between the two clusters [11, 12]. In addition, the study analyzed the correlation between HPV infection and primary bladder tumor disease, and the results showed that there is no correlation between the expression of HPV-16 and the degree of tumor differentiation and age of patients (*P* > 0.05). The results of this study are consistent with other research results. Sex is not upper, which is related to the pathological composition and case conditions [13, 14]. However, HPV-16 has upper sensitivity and specificity for judging the expression and cell and molecular deletion of primary bladder tumors, and the results suggest that HPV-16 can be used as an important basis for judging disease progression [15, 16]. The analysis of the expression status of HPV-16 in primary bladder tumors can more accurately follow-up and grasp the prognosis of patients. The prognosis analysis showed that there were 57 patients, including 11 patients with single tumor and 46 patients with multiple tumors. After 3 years of continuous follow-up, 37 situations of tumor-free survival, 17 situations of recurrence, and 3 situations of death were found during follow-up. The results confirmed that HPV-16 can be used as an important reference for patient prognosis analysis [17, 18].

Research on the expression of HPV-16 in primary bladder tumors and the analysis of the loss of cell differentiation can provide theoretical reference value for the judgment of disease status [19, 20]. Even so, this study only analyzed the correlation of the expression of HPV-16. The lack of completeness of the research content will affect the accuracy and rationality of the research to a certain extent. Therefore, further analysis and exploration are required to ensure the feasibility of the study [21].

## 5. Conclusion

HPV-16 is an upper, expressed in primary bladder tumors and participates in cell differentiation and deletion. It may provide effective guidance and basis for the diagnosis of primary bladder tumors. It is an important factor in judging the pathological stage and prognosis of patients, and can be used for healing measures to provide theoretical reference.

## Figures and Tables

**Figure 1:** Analysis of HPV subtypes in patients. Note: HPV-6, HPV-16, HPV-18, HPV-26, HPV-39, HPV-45, HPV-51, HPV-53, HPV-56, HPV-59, HPV-66, and HPV-68. The proportions of HPV-82 subtypes were 10.71%, 28.57%, 17.86%, 3.57%, 7.14%, 3.57%, 3.57%, 7.14%, 3.57%, 3.57%, 3.57%, 3.57%, and 3.57%, respectively.

**Figure 2:** Analysis of tumor stage in two clusters of patients (situations, %). Note: the percentage of stage 1, a, and 2a staging in the HPV-related cluster was 32.14%, 35.71%, and 32.14%, respectively, and the percentage of stage 1, a, and 2a staging in the HPV-unrelated cluster was 27.59%, 34.48%, and 37.93%, respectively.

**Figure 3:** Analysis of postoperative pathological expression in two clusters of patients. Note: the postoperative pathological upper and bottom expression rates of the HPV-related cluster were 60.71% and 37.93%, respectively, and the postoperative pathological upper and bottom expression rates of the HPV-unrelated cluster were 37.93% and 72.41%, respectively.

**Figure 4:** The value of HPV-16 in judging primary bladder tumor expression and cell and molecular deletion. Note: HPV-16 has upper sensitivity and specificity in judging the expression of primary bladder tumors and the deletion of cellular molecules. The results suggest that HPV-16 can be used as an important basis for judging disease progression.

**Figure 5:** Analysis of patient prognosis. Note: the proportions of patients with single tumor and multiple tumors were 19.30% and 80.70%, respectively, and the tumor-free survival, recurrence, and mortality of patients were 64.91%, 29.82%, and 5.26%, respectively.

**Table 1:** Analysis of HPV subtypes in patients (situations, %).

Subtype	Number of detections (example)	Infection rate (%)
HPV-6	3	10.71
HPV-16	8	28.57
HPV-18	5	17.86
HPV-26	1	3.57
HPV-39	2	7.14
HPV-45	1	3.57
HPV-51	1	3.57
HPV-53	2	7.14
HPV-56	1	3.57
HPV-59	1	3.57
HPV-66	1	3.57
HPV-68	1	3.57
HPV-82	1	3.57

**Table 2:** Analysis of tumor stages in two clusters of patients (situations, %).

Tumor stage	HPV-related clusters (*n* = 28)	HPV-unrelated cluster (*n* = 29)	*X* ^2^	*P*
Stage 1	9 (32.14)	8 (27.59)	0.024	0.886
Stage a	10 (35.71)	10 (34.48)		
Stage 2a	9 (32.14)	11 (37.93)		

**Table 3:** Analysis of postoperative pathological expression in two clusters of patients (situations, %).

Postoperative pathology	HPV-related clusters (*n* = 28)	HPV unrelated cluster (*n* = 29)	*X* ^2^	*P*
Upper expression	17 (60.71)	11 (37.93)	0.889	0.346
Bottom expression	7 (25.00)	21 (72.41)		

**Table 4:** Analysis of general data of patients.

General information	HPV-related clusters (*n* = 28)	HPV-unrelated cluster (*n* = 29)	*X* ^2^	*P*
Age (years)	61.46 ± 3.58	63.10 ± 3.29	1.802	0.077
Sex (male/female)	21/7	21/8	7.000	0.008
Alcohol consumption			1.636	0.201
Regular daily drinker	20 (71.73)	14 (48.28)		
Occasionally/never	8 (28.57)	15 (51.72)		
Smoke or not				
Smoke	16 (57.14)	11 (37.93)	2.643	0.267
Have quit smoking	7 (25.00)	8 (27.59)		
Never	5 (17.86)	10 (34.48)		

**Table 5:** Correlation analysis of HPV-16 expression with tumor differentiation and age in patients.

General information		HPV positive (*n* = 28)	HPV negative (*n* = 29)	*X* ^2^	*P*
Age (years)				1.709	0.425
<65	28	9 (32.14)	19 (67.86)		
65~74	24	11 (45.83)	13 (64.17)		
≥75	5	1 (20.00)	4 (80.00)		
Degree of differentiation					
Upper differentiation	6	2 (33.33)	4 (66.67)	1.417	0.492
Moderately differentiated	24	6 (25.00)	18 (75.00)		
Bottom differentiation	27	11 (40.74)	16 (59.26)		

## Data Availability

The dataset used in this paper are available from the corresponding author upon request.
